This article has been retracted.

# Exploration of Strategies for Organic Integration of Labor Education and Occupational Therapy for College Students

**DOI:** 10.1155/2022/7115412

**Published:** 2022-07-21

**Authors:** Linna Du, Weizheng Wang

**Affiliations:** ^1^School of Harbin Normal University, Harbin, Heilongjiang 150025, China; ^2^School of Mudanjiang Normal University, Mudanjiang, Heilongjiang 157011, China

## Abstract

This paper analyzes the actual functions of the labor education and occupational therapy phase through an in-depth study of labor education and occupational therapy for college students and explores the strategies of organic integration of labor education and occupational therapy for college students. This paper carries out a holistic theoretical construction of labor education in schools and systematically analyzes the components of labor education objectives in colleges and universities, labor education contents in schools, labor education implementation in schools, and labor education evaluation in schools. The main goal of labor education in colleges and universities is to guide students in establishing a scientific concept of labor and constructing a labor education resource system. It focuses on strengthening the construction and improvement of the labor education theoretical system, promoting the construction of labor education disciplines and professional courses, and attaching importance to the training of labor education teachers in the new era to contribute to the perfection of labor education. The system of labor education practice should be innovated. Of course, the labor practice activities based on institutionalization should be implemented. The cycle of labor activities based on the principle of continuity should be strengthened, and the effectiveness of labor education should be improved totally from explicit and implicit instructions. The core of occupational therapy is to help college students adapt to social work, give full play to their self-worth, obtain economic resources, and improve self-confidence. The organic integration of labor education and occupational therapy shows that it can help students ease their social adaptability and adapt to social functions, improve the reemployment rate, and improve students' overall health. Therefore, the practical research on labor education and occupational therapy should be strengthened.

## 1. Introduction

Labor forms are constantly iterating and changing, and workers, labor tools, and labor objects have all undergone fundamental changes and society's development. In this context, integrating labor education into the school education system is one of education reform's core issues [1]. Human beings have accumulated endless knowledge and skills during the long historical process, covering a wide range and deep capacity. It is difficult for school education, which aims to achieve universal education, to teach all these knowledge and skills, and students cannot afford their learning capacity. Therefore, dividing knowledge and skills into categories so students can learn systematic knowledge and skills is an integral part of educational reform and development. In this way, routine, basic, and specialized knowledge and abilities, classified in the sea of knowledge and skills, are gradually constructed in “disciplines” in educational practice [2]. According to different knowledge and skill characteristics, the subjects are given specific educational objectives, educational contents, implementation, evaluation, and other elements, forming the corresponding subject curriculum theory. The integration of labor education into the school education system emphasizes the design and arrangement of subjects with “labor” as the core. In this discipline, “labor” is not only the goal of education but also the content of education, which is education about labor, and the way of education and teaching, which is education in labor [3]. In the new era, labor education in schools has profound connotations and value implications of the times. Only by promoting the theoretical construction of labor education in schools, making overall design and scientific planning of labor education in schools, and focusing on improving the system of labor education in schools can we effectively apply the objective historical law of “combining education and production work” in the modern education system. Only by bridging the transformation of labor education in the theoretical form to labor education in its natural state can we realize the scientific, holistic, and dynamic change of labor education theory to labor education practice in schools, and only then can we answer the new questions raised by labor education practice with the latest labor education theoretical achievements and thus promote the overall development of human beings and the overall progress of society [4]. Therefore, it is of great theoretical significance to take labor education in schools as the research object, explore the characteristics and laws of labor education in schools in-depth, and systematically construct a theory of labor education in schools containing educational objectives, educational contents, and educational content implementation and educational evaluation.

Labor education in colleges and universities has developed into a new era, and its function of nurturing people has been gradually enhanced. However, the current practice of labor education in colleges and universities still suffers from the fundamental dilemma of hindered development; i.e., the high demand for labor education in colleges and universities in social development contradicts the weak supply of labor education effect in colleges and universities, which provides a breakthrough for research [5]. However, no matter how history changes, labor education in colleges and universities still maintains its unique value. It is necessary to conduct research on labor education in colleges and universities. Meanwhile, the promulgation of policies related to labor education in colleges and universities also provides a strong impetus for the research. With the stable and continuous development of higher education, the employment competition for college graduates is becoming more and more fierce. Employers have put higher requirements on students' labor operation skills and practice ability. Hence, colleges and universities play an essential role in educating students to correct their labor cognition, enhance their labor operation skills, and improve their labor practice ability [6]. However, labor education in colleges and universities has been gradually neglected. News about poor independence of college students, good and bad work, and low vision have been reported from time to time. The problems reflected by these phenomena deserve our deep consideration [7]. The issues that college students do not clearly understand labor education and insufficient labor operation ability cannot be ignored. Therefore, there is an essential breakthrough in the research on the problems and countermeasures of labor education practice in colleges and universities; that is, the contradiction between the lack of labor education in colleges and universities and the demand of society for labor education in colleges and universities is becoming more and more prominent. Labor education can help college students build a good personality, sharpen a strong will, and refine a noble character. Colleges and universities should consider the actual situation and start from three aspects, ideological leadership, personal practice, and organic integration, and actively build an education system for college students with comprehensive development of moral, intellectual, physical, aesthetic, and labor.

Occupational therapy uses specific activities to assist in the recovery of various physical or psycho-psychological disorders and alleviate and soothe students' developmental or social dysfunctions to achieve maximum independence in life [8]. This paper explores the sense of organic integration of labor education and occupational therapy for college students, which can help them adapt to social functioning, increase their confidence in facing environmental challenges, enhance their social adjustment, strengthen their self-identity, and promote the normalization of social life [9]. Some scholars believe that after occupational therapy, students' social adjustment ability scale scores and daily living ability scale scores have been improved, suggesting that college students' self-care ability has been improved, their interest in things has increased, and they can communicate with others more effectively; their initiative has been strengthened, their interpersonal skills have been exercised, and their social function is close to normal. Regarding social function restoration, scholars are more consistent in their conclusions that occupational therapy can improve students' positive emotions, expand social support, strengthen students' verbal and emotional communication with others, and reduce the degree of emotional indifference [10]. There was a significant improvement effect on the social adjustment of college students who had just joined the workforce.

## 2. Related Works

In the long history and reality, people have long recognized the critical role of labor in society and life. They also know that labor education has strong practicality in talent training and helps students cultivate good qualities [11]. The combination of labor and education makes the two promote each other and develop together. However, during the development of primary education, in the long run, labor education for students has always been neglected compared to their academic performance, and there are still problems in its implementation on paper [12]. As primary education enters a new era, labor education has received more and more attention from the education sector to realize moral education as one of the essential contents of talent cultivation. Heinrich and Green believe schools, rather than families, should be responsible for labor education in the new era [13]. Regardless of whether this view is biased, schools are rightly accountable for providing labor education to students, playing an irreplaceable role in cultivating students' correct concepts of labor and their awareness of active participation in labor. Schools can also easily elevate students' positive group labor phenomenon to a universal social value to be promoted. The traditional way of labor education can inadvertently be separated from the intention of labor education, losing the spiritual weight given by labor and turning the process of labor education into mere physical work. In contemporary labor education, we should avoid this situation as much as possible and look at labor education with an integrated mindset, combining “body and brain,” labor and spirit. The content and form of labor education are inadequate because of the pressure of high school studies and the need to consider more factors when conducting labor education [14]. After communicating with front-line teachers of various subjects in secondary schools, I found that biology, because of its unique characteristics related to life production and life activities, can help guide students to carry out productive work through the rational use of biology knowledge, so the biology classroom is an excellent new channel for labor education compared with other subjects.

There are few conceptual definitions of labor education in colleges and universities; most of them are about labor education, and there is not yet a clear consensus. The abstract description of labor education is mainly divided into two categories: one considers labor education a kind of educational content, and the other considers labor education a literary form [15]. In terms of labor education as content, college students should establish correct labor values, form fundamental labor dynamics, improve their quality of life and proficiency in labor skills, develop good labor habits, and enhance their passion for labor. As a form of labor education, labor education is just a means to cultivate students' overall moral, intellectual, physical, aesthetic, and labor development [16]. Through labor education, college students can participate in various practical activities to exercise themselves, thus realizing the evolution of morality, intellect, physique, aesthetics, and labor. The study found that the previous conceptual definition of labor education mainly focuses on the following. Some experts think labor education is a kind of activity. Metzger and Duening think labor education is primarily an activity that takes college students as the main body of action and carries out activities to cultivate college students to establish correct labor values [17]. Mathews et al. believe that labor education is a practical activity that leads people to return to their true nature [18].

Occupational therapy is an advanced treatment technique widely used to restore or maintain individuals and play a pivotal role in their future development [18]. The main areas of occupational therapy are home care skills and self-care training, work skill training, social guidance, and study guidance. There is a relative lack of application and research in occupational therapy in higher education, especially for college students. Since establishing the School Services Section, we have developed student case management services in colleges and universities [19]. We conducted occupational therapy with students in the student case management service and made a controlled study to observe its effect on rehabilitation outcomes. Occupational therapy is a psychosocial treatment method that helps students with stable symptoms train work and social skills, provide employment opportunities, help students maintain their career development, gain income from work, train skills, increase confidence, improve quality of life, and achieve therapeutic goals [20]. The result of occupational therapy is different from simple labor, and the training of students is skillful and vocational, emphasizing returning to society. Its development can be divided into traditional occupational therapy and supported employment. Conventional occupational therapy includes sheltered employment, transitional employment, skills training, day treatment, and occupational clubs [21]. Traditional occupational therapy advocates providing students with prevocational education and then helping them return to work. Conventional occupational therapy has been carried out earlier and has been reported to help college students improve their skills and self-confidence, gain financial resources, and reduce relapse rates, and after long-term follow-up, it is believed that traditional occupational therapy can help students obtain competitive jobs. However, some scholars believe such methods do not significantly increase students' employment rates.

## 3. Analysis of the Organic Integration of Labor Education and Occupational Therapy for College Students

### 3.1. Theoretical Analysis of Labor Education and Occupational Therapy for College Students

The individual function of labor education in schools refers to the objective influence on education. Labor is the basis for the survival and development of human beings and human society because labor produces material means of living and social relations and human beings themselves. In labor, the individual must deal with the relationship between man and nature, man and society, and the relationship between man and his development. In this process, human beings achieve the comprehensive development of their working ability, social relations, and free personality [22]. Labor education in school educates people through “labor,” pointing to the all-round development of students, guiding them to achieve the all-round development of labor ability in dealing with the relationship between human beings and nature, the all-round development of a social relationship in dealing with the relationship between human beings and society, and the all-round development of free personality in dealing with the relationship between human beings and their development. Labor education in school is conducive to guiding students to realize the comprehensive development of labor ability in labor. The overall effect of human labor ability includes both physical growth and intellectual development. Occupational therapy refers to the purposeful engagement in some occupational training designed to restore motivation, confidence, and specific skills for treating physical or mental impairments. Rehabilitation is a form of treatment that promotes the return to normal or near-normal physical and psychological dysfunction or disability caused by injury, disease, developmental defects, and other factors. It is an essential part of rehabilitation medicine. The reform and opening, under the guidance of the policy of “science and technology is the first productive force,” have accelerated the effect of “intellectual” education in terms of depth and breadth, but this has led to the development of “mental labor” and “physical labor” of students. However, this has severely imbalanced students' “mental” and “physical” work. The implementation framework of labor education is shown in Figure 1.

Labor education in schools is conducive to guiding students to realize the comprehensive development of their free personality in labor. The entire story of human free character, i.e., promoting human independence, conscious initiative, and creativity, is the core embodiment and highest goal of comprehensive human development. To achieve this, we must continue to transcend ourselves and pursue the complete story of our free personality. The youths are currently confined in the “iron wall” school, buried in test knowledge, personality suppression, and thinking solidification. There are phenomena such as good and bad work, desire to get something for nothing, blind consumption, and commodity fetishism. The modern life dominated by information technology is also full of the “lack of subjectivity” and the “spiritual homeland nowhere to be found.” In this context, school labor education can guide students to experience the value and joy of life in labor practice, to show their will in the labor process experience, and to realize their self-worth in the sharing of the fruits of labor, which is conducive to the comprehensive development of students' free personality in delivery.

With the popularization of the Internet and the massive use of cell phones and computers, the ways and means for college students to learn about society have greatly expanded. They can get the latest news and knowledge worldwide through microblogs and web news anytime and anywhere. But this kind of information data is only “seen” through our eyes. We cannot ensure the accuracy and objectivity of the information, nor can we give the students a “brain-made real world” just by using such online details. Labor originates from the needs of life, and work means that college students should touch the entire society with their hands and experience it with their feet. To maintain the daily activities of survival, we need to master some daily living skills so that the real world can react closely. Moreover, college students have expressed willingness to participate in family work; 9% are very active, 58% are involved in family work, and 22% have negative emotions. As shown in Figure 2, most college students have a positive attitude toward household work and want to learn more life skills.

Traditional occupational therapy places more emphasis on the psychological and symptomatic stability of college students and on the gradual development of workability, with the drawback that skills cannot be evaluated from actual work, and the institutions providing occupational therapy are generally scattered and independent, which is not conducive to continuous support and follow-up. It is worth noting that the issue of job setting and operation participation, we grasp the principle that according to the actual situation of students, physical ability, interests, strengths, and individual differences to arrange suitable positions, more conducive to exploring the average psychological potential of students. The idea of “placement training” is different from the traditional occupational therapy approach. It has the advantage of helping college students find jobs in the first place, emphasizing rapid employment, with employment as the primary goal, considering college students' personal preferences and strengths, and integrating labor education and occupational therapy [23]. Occupational therapy is combined to provide services, and it is easy to maintain long-term support. Supported employment achieved higher employment rates for college students just entering society, with significantly better hours and wages than traditional occupational therapy modalities. No empirical studies show that supported employment leads to more significant stress and higher unemployment rates. This suggests that supported employment has tremendous advantages in helping college students get jobs. Workforce education needs to rely not only on the “words” of faculty and staff but also on the “example” of faculty and staff. All staff members must pay attention to labor education from the ideological point of view and fully realize the importance and necessity. All staff members should clarify their roles and tasks in labor education and master the ways and methods of labor education. All teaching staff has the concept of the labor education system. During the treatment period, students are asked and encouraged to engage with their surroundings to stimulate their interest, confidence, and courage in life and work and to continue to gain experience. They can not only complete their work in labor education but also consider the overall situation and continuously explore the labor education elements that adapt to the characteristics of the times, meet students' needs, and guide their interests to form an educational synergy with the participation of all staff.

### 3.2. Strategy Design for the Organic Integration of Labor Education and Occupational Therapy for College Students

Labor education in schools promotes the social ethos of labor happiness. Unlike purely intellectual or general education activities in the broad sense, labor education in schools is a specialized curriculum for national education. Its essence is a practical activity cultivated by the Marxist concept of labor. From the perspective of its essential attributes, labor education has the scientific characteristics that other curricula generally have. At the same time, it must have political values that additional education does not have or is not significant. Labor education in schools adheres to its ideological orientation, realizes the organic unity of scientific and political rationality, disseminates, cultivates the Marxist concept of labor, and helps promote the social ethos of labor happiness. All faculty members have the idea of a labor education system. They can accomplish their own work in labor education. Still, they can also consider the overall situation and continuously explore the labor education elements that adapt to the characteristics of the times, meet the needs of students, and guide their interests, to form an educational synergy with the participation of all staff members.

On the one hand, labor education in schools guides future workers to revere labor and love labor. Young people's labor concept has changed dramatically in developing a socialist market economy, facing the contradictions between labor and capital, labor and knowledge, and labor and acquisition. Some young people have the mentality of excellent and insufficient labor, desire to get something without working, blind consumption, and commodity fetishism. School labor education guides young people to establish correct labor values, which is conducive to helping them understand that labor is a source of happiness and discard the unwanted thoughts of good and bad labor and gain without work. On the other hand, in the historical background of globalization, informatization, and networking, western social trends such as altruism, egoism, and consumerism are prevalent. Some young people are caught in a conflict of values, with a distorted and misplaced worldview, outlook on life and values, abandoning or even opposing Marxist beliefs [24]. Extreme individualism and utilitarianism reflect the lack of faith of some youths, especially their insufficient understanding of the Marxist concept of labor. In the era of multiculturalism, school labor education insists on cultivating the Marxist view of labor, which is conducive to correcting the social climate; enabling students to establish the value of labor as the most glorious, noble, great, and beautiful; and inspiring them to create happiness with labor in the future and become hardworking, honest, and creative laborers. The design of the labor education curriculum for college students in higher education is shown in Figure 3.

The cultivation of labor skills and the establishment of labor values need to be realized in labor practice. Whether in family education, parents teach their children by example; in school education, teachers teach them by example; or in social education, seniors give detailed guidance; all communicated through symbolic and physical language between people. Labor education focuses on practice, and when college students choose their favorite type of labor, 84.38% of them choose public welfare labor on campus, 78.13% choose top-notch work, and 84.38% choose employment practice labor, which shows that college students prefer labor education through the way of in-depth communication with people and society. It is easier for us to gain new knowledge and help from others in specific social situations to build our advantages. Practical labor activities for college students do not stop at simple volunteering, such as mechanical labor like sweeping floors and wiping tables, but rather complex work that requires the interplay of mental and physical strength. This is because professional advice is not only better for college students to learn more knowledge and better participate in labor practice activities. It also makes college students feel the regularity and professionalism of the organizers and believe that this activity is beneficial to their development. The considerations of college students' participation in labor practice activities are shown in Figure 4.

A curriculum is a basic form of implementing labor education, and improving the structure of the labor education curriculum is an important measure to enhance the effectiveness of labor education [25]. The “Trinity” labor education curriculum system is based on China's actual situation and objective education laws. As shown in Figure 5, we should establish the implementation standards of labor education curriculum, make macro regulations on the structure of labor education curriculum based on the primary national conditions and education laws, and try to make labor education have rules to follow. On this basis, we will promote the coordination of the national curriculum, local curriculum, and school-based curriculum at the management level and form an organic whole consisting of the primary curriculum, extension curriculum, and creative curriculum, as well as an integrated curriculum structure consisting of explicit curriculum and implicit curriculum.

## 4. Analysis of Results

### 4.1. Analysis of Labor Education and Occupational Therapy Model for College Students

Artificial intelligence is applied as a new tool in labor education teaching. According to the habits of college students' learning courses, personalized design is made to realize the excellent management of college students, unique learning plans are made for college students according to the data results, and labor education in colleges and universities achieves innovative development. They guide college students to use smart devices to independently prestudy labor courses. The professional guidance is not only better for the students to learn more knowledge and better participate in the labor practice activities. It also makes the students feel the regularity and professionalism of the organizers and believe that this activity is beneficial to their development. We organized college students to participate in social service labor in their free time to strengthen college students' experience and cognition and recognition of specific work in the operation of knowledge and action and internalize such feelings to realize the cultivation goals of college students' labor concept, labor spirit, labor ability, and quality. Teachers in colleges and universities set up virtual labor scenes in the classroom and use multimedia to display the textual interpretation of labor and vivid cases in a dynamic form. The school learning of labor education can relate to the case materials. The effectiveness of labor education and classroom connection can be enhanced. To enhance college students' recognition of labor, let the value of work into their minds to achieve transformation. For example, set up labor courses and lead students to precourse prestudy and independent study. Guide them to learn to share, exchange, review, and consolidate in cooperation, and change students' knowledge construction mode. Colleges and universities should offer AI intelligent labor courses, relying on laboratories to give education targets a more comprehensive and systematic understanding of the techniques and laws of agricultural production. The primary data analysis on labor education is shown in Figure 6.

Build a digital curriculum system for labor education. The use of virtual reality technology creates a new educational, ecological environment for the development of labor education, provides an environment and collaborative partners to support the labor learning of college students, enables them to complete labor tasks through controlled “virtual reality” operations, and then obtains a comprehensive understanding and “embodied” experience of labor. The “virtual reality” operation enables college students to complete labor tasks through controlled “virtual reality” operations, thus gaining a comprehensive understanding of labor and “embodied” emotional experience. Colleges and universities fully play the technical advantages of artificial intelligence to build digital, video, and virtualized labor culture courses, labor practice courses, and labor fun courses. Design feasible labor education plans according to college students' physical and mental development characteristics, uses campus resources, and combines with school characteristics to offer new medicine and environmental science courses [26]. Combine with AI common labor, organize college students to participate more in labor practice so that college students can get close to AI and feel the latest achievements of human wisdom. In the era of artificial intelligence, we should aim at intelligent integration of labor education content, intellectual development of labor education practice, and smart enhancement of labor education elements and improve the effectiveness of labor education in colleges and universities by converting the cognitive mode of labor education, insisting on the humanistic heritage of labor education, and clarifying the technical boundary of labor education.

Teach entrepreneurship in the process of carrying out labor education activities. Colleges and universities should carry out education on career planning for hit students, cultivate college students' career interests, and enable them to form correct concepts of labor and life goals. Colleges and universities should strengthen innovation and entrepreneurship education to improve the employment rate of college graduates. Colleges and universities invite famous scholars, excellent entrepreneurs, and model workers to offer entrepreneurship practice courses for teachers and students. At the same time, colleges and universities should add labor education-related content such as career cognition, career characteristics, employment outlook, and entrepreneurial outlook to the innovation and entrepreneurship courses and offer courses on innovation and entrepreneurship elements and general education courses on basic labor knowledge and practical education. Understanding how to apply for starting a business and business organization and management is taught during lectures. College students are guided to participate in innovative labor education and training to enhance their labor awareness effectively. The organic integration of labor education and occupational therapy for college students is explored in the sense that occupational therapy can help them adapt to social functions, improve their confidence in facing environmental challenges, enhance social adaptation, strengthen their self-identity, and promote normalization of social life. Colleges and universities take the initiative to assume the functions of teaching labor skills, cultivating labor values and career education, helping college students know how to revere and respect labor in labor education, enhancing their emotions for working people, developing their awareness and habits of loving delivery, and finding beauty in struggle and experiencing beauty in respecting labor. The practical test of labor education in school is shown in Figure 7.

Establish a professional team of teachers to carry out labor education. Firstly, introduce model workers into the campus in colleges and universities, thus realizing the cultivation of labor value education and entrepreneurial consciousness education. Secondly, colleges and universities should build labor education and occupational therapy teachers with a broad vision and profound theoretical attainments. Occupational therapy and labor education have certain similarities; strengthen school-enterprise cooperation and integration of production and education; reform teachers in various aspects such as assessment, training, and treatment; maintain the work enthusiasm of the teacher team; encourage teachers of professional courses to drive student groups to go deeper into front-line practice; and strengthen labor education and innovation and entrepreneurship education. The combination of labor education and innovation and entrepreneurship education is promoted.

Occupational therapy is carried out in the process of labor education. Colleges and universities combine excellent labor culture with labor education practice by organizing occupational therapy lecture series and innovative and entrepreneurial work design competitions [27]. Colleges and universities organize and mobilize college students to participate in various technical exchange competitions, such as vocational skill competitions, to cut skills and scientific research to improve the technical level and enhance the vocational honor of labor. Colleges and universities help college students establish the concept of innovation and entrepreneurship education that integrates the shaping of labor values with the cultivation of innovative thinking, entrepreneurship, and creative ability. Universities hold innovation and entrepreneurship competitions with labor education as the mainline and set up “public welfare labor entrepreneurship project group,” “labor creativity project group,” “labor education practice demonstration project group,” etc. To guide college students to respect labor, let them understand that work is the most glorious, inspire them to participate in innovation and entrepreneurship, and motivate them to create value and shape their lives in labor.

### 4.2. Labor Education and Occupational Therapy for Students in Higher Education Organic Integration of Strategies for the Realization

According to the analysis, occupational therapy refers to the application of relevant knowledge of human development, psychology, behavioral therapy, learning theory, and system theory to help college students meet their needs, increase their self-knowledge ability, establish a correct outlook on life and values, cultivate life skills and leisure hobbies, and establish regular living habits. The study also is aimed at improving social skills and promoting good work attitude and workability [28]. In this study, negative PANSS scale symptom scores, general college student scores, total scores, ADL, social skills, and social adaptive functioning scores decreased after labor education and occupational therapy compared to preintervention, and the difference was statistically significant (*P* < 0.05) and also significantly decreased compared to preintervention, and the difference was statistically significant (*P* < 0.05); scores increased dramatically compared to preintervention, and the difference was statistically significant (*P* < 0.01) and also significantly increased compared to nonorganic integration, with a statistically significant difference (*P* < 0.01). This indicates that occupational therapy has improved the social adjustment of college students and cognitive aspects and has improved the students' ability to perform daily life and adapt to social life through assistance and various rehabilitation services. Students engaged in learning job skills through this low-stress, noncompetitive work, which is an essential step towards open employment, significantly increased organic integration employment compared to the absence of labor education. This suggests that students who participated in occupational therapy had stress resistance when participating in work. The decrease in all PANSS scores and students' daily living skills, social skills, and social adjustment without training may be related to students' maladjustment. In summary, occupational therapy in sheltered employment for college students can help them improve their social adjustment, self-care, and problem-solving skills; maximize their overall training; and positively impact their integration into society and employment. The analysis of occupational therapy data of students in higher education is shown in Figure 8.

There were highly significant differences (*P* < 0.01) in SRCP total score, negative factor score, and NOSIE total score and significant differences (*P* < 0.05) in affective factor score when comparing before and after occupational therapy training for college students. SRCP total score, negative factor score, and affective factor score were not significantly different from those three months after the workout. NOSIE was significantly different between before and three months after the training. Significant differences were found between NOSIE before training and three months after training. The above results suggest that specific effects emerged after job occupational function training. The results indicated that their negative and affective symptoms showed a slower time to effect, which was estimated to be related to the degree of labor education, consistent with the reports of related studies. Because the postoccupational training in this paper was compared with the generally reported group work therapy, a closed management operation in schools, these students' present experimental training procedure emphasized the incentive mechanism of using normal psychological activities. The postoperation was competitively performed, and the whole training was openly managed inside and partly outside the institution. The students strengthened their verbal and emotional communication with each other during the induction and leisure time. As a result, the students enhance their oral and dynamic communication with each other during their work and leisure time, which reduces their emotional indifference and promotes their mental, social, and physical functions and their ability to adapt to social life. As for the adaptability to student work, there was no significant difference before and after the training. It is worth noting that the principle of job setting and participation is to arrange suitable jobs according to the students' actual situation, physical ability, interests, strengths, and individual differences, which is more conducive to the development of the students' average psychological potential. The before-and-after comparison of the organic integration of labor education and occupational therapy is shown in Figure 9.

The direction and path of the organic integration of labor education and occupational therapy education for human development create good preconditions for the deep integration of both. Students in colleges and universities should deeply understand the consistency of labor education and occupational therapy goals. They should take labor education as an essential direction for implementing vocational education in colleges and universities and vocational education as a necessary labor education. Colleges and universities should accelerate occupational therapy education cultivation goals to cultivate students' labor spirit. Occupational therapy education is based on labor value and focuses on shaping students' entrepreneurial spirit of daring to start up, innovation, and hard work. Realizing that labor education gives strong support to occupational therapy education guarantees that labor education follows the trend of the times, transforms into intellectual and creative labor, liberates the labor force, and promotes occupational therapy education to create more social benefits.

## 5. Conclusion

As the future force of social construction, students in colleges and universities are responsible for the great mission of national rejuvenation. In the new era, strengthening labor education for college students helps cultivate red and professional college students with morals and talent. It has irreplaceable significance to the construction and development of an innovative country. Admittedly, as labor education for college students has received more and more attention, academic research has also increased in recent years, and specific educational results have been achieved. However, under the influence of many realistic circumstances, there are still some problems, and labor education for college students is hindered. To build a platform for labor education practice, put labor education into practice and produce results, these things need the cooperation of society, families and college students. Make full use of social resources such as labor education practice bases and innovation bases of industry-university-research cooperation, combined with study trips and professional internships, etc., to deepen college students' perception, experience, and reflection on the current occupational needs of labor in various industries; help them gain initial occupational impressions; gradually cultivate the spirit of hard work and perseverance in labor exercises; and lay a solid foundation for entering society and going to work in the future. We should build a labor education and occupational therapy community with the linkage of general and vocational education. Focus on labor experience to promote the formation of basic labor skills and vocational literacy to lay the foundation for college students' career development and life happiness. Labor education in colleges and universities has different forms and characteristics in other contexts, which to a certain extent indicates that research in this area is a long-term and continuous work. We will continue to study and improve the shortcomings of this study in the future.

## Figures and Tables

**Figure 1:** Framework for implementing labor education.

**Figure 2:** Attitudes of college students' participation in labor education.

**Figure 3:** Design of labor education curriculum for college students.

**Figure 4:** Considerations of college students' participation in labor practice activities.

**Figure 5:** Structure of labor education in university schools.

**Figure 6:** Analysis of the primary data of labor education.

**Figure 7:** School labor education practice test.

**Figure 8:** Analysis of occupational therapy data for college students.

**Figure 9:** Comparison before and after organic integration of labor education and occupational therapy.

## Data Availability

The data used to support the findings of this study are available from the corresponding author upon request.

## References

[1] Eryong X., Li J. (2021). What is the ultimate education task in China? Exploring “strengthen moral education for cultivating people” (“Li De Shu Ren”). *Educational Philosophy and Theory*.

[2] Jaegers L. A., Dieleman C., Dillon M. B., Rogers S., Muñoz J. P., Barney K. F. (2020). Justice-based occupational therapy initiative: advancing occupational justice in criminal justice systems. *Annals of International Occupational Therapy*.

[3] Parsons A. F. (2020). Exploring everyday chemistry: the effectiveness of an organic chemistry massive open online course as an education and outreach tool. *Journal of Chemical Education*.

[4] Tsai M. C., Shen P. D., Chen W. Y., Hsu L. C., Tsai C. W. (2020). Exploring the effects of web-mediated activity-based learning and meaningful learning on improving students’ learning effects, learning engagement, and academic motivation. *Universal Access in the Information Society*.

[5] Yin J., Tang F., Zou L. (2021). Research on the “otse” mode of classroom cultivation of teacher students’ professional quality based on the concept of cooperative learning. *Advances in Educational Technology and Psychology*.

[6] Gkonou C., Miller E. R. (2021). An exploration of language teacher reflection, emotion labor, and emotional capital. *TESOL Quarterly*.

[7] Li X., Wang W. (2021). Exploring spatial cognitive process among STEM students and its role in STEM education. *Science & Education*.

[8] Iyamuremye A., Mukiza J., Nsabayezu E., Ukobizaba F., Ndihokubwayo K. (2022). Web-based discussions in teaching and learning: secondary school teachers’ and students’ perception and potentiality to enhance students’ performance in organic chemistry. *Education and Information Technologies*.

[9] Hansen A. K., Langdon T. R., Mendrin L. W., Peters K., Ramos J., Lent D. D. (2020). Exploring the potential of 3D-printing in biological education: a review of the literature. *Integrative and Comparative Biology*.

[10] Tom J. W., Green R. A., Cherney E. C., Huang M., Lott J. (2022). Empowering women in chemical sciences and engineering through outreach: a platform to explore careers in the pharmaceutical industry. *Journal of Chemical Education*.

[11] Pérez-Eransus B., Martínez-Virto L. (2020). Social work education in Spain: evaluation and challenges for a new generation of social workers. *Social Work Education*.

[12] Xue E., Li J., Li T., Shang W. (2021). China’s education response to COVID-19: a perspective of policy analysis. *Educational Philosophy and Theory*.

[13] Heinrich W. F., Green P. M. (2020). Remixing approaches to experiential learning, design, and assessment. *The Journal of Experimental Education*.

[14] Gustafson E. L., Lakind D., Walden A. L., Rusch D., Atkins M. S. (2021). Engaging parents in mental health services: a qualitative study of community health workers’ strategies in high poverty urban communities. *Administration and Policy in Mental Health and Mental Health Services Research*.

[15] Edwards B. M., Cameron D., King G., McPherson A. C. (2021). Contextual strategies to support social inclusion for children with and without disabilities in recreation. *Disability and Rehabilitation*.

[16] Steele P., Burleigh C., Bailey L., Kroposki M. (2020). Studio thinking framework in higher education: exploring options for shaping immersive experiences across virtual reality/augmented reality curricula. *Journal of Educational Technology Systems*.

[17] Metzger M. L., Duening T. N. (2021). Exploring the use of virtues to facilitate identity construction among management students. *European Management Journal*.

[18] Mathews M., Ryan D., Buote R., Parsons S., Lukewich J. (2020). A qualitative study exploring the influence of clinic funding on the integration of family practice nurses in Newfoundland and Labrador. *Nursing Open*.

[19] Hart A., Psyllou A., Eryigit-Madzwamuse S. (2020). Transitions into work for young people with complex needs: a systematic review of UK and Ireland studies to improve employability. *British Journal of Guidance & Counselling*.

[20] Dunne M., Nisbet G., Penman M. (2021). How speech pathology educators conceptualise reflection in practicum contexts influences student learning experiences. *Reflective Practice*.

[21] Ramsey C., Ricket A. (2020). Examining physical space, leadership inheritance, and “authentic” community engagement through co-constructed autoethnography. *American Journal of Qualitative Research*.

[22] Meng S., Tao F., Han L. The Joint Development of College Labor Education and Quality Education Based on the New Era.

[23] Mastel-Smith B., Kimzey M., Garner J., Shoair O. A., Stocks E., Wallace T. (2020). Dementia care boot camp: interprofessional education for healthcare students. *Journal of Interprofessional Care*.

[24] Pope R. J., Jones J. N. (2020). Exploring organizational strategies and participant experience in the young adult diversion court. *Victims & Offenders*.

[25] Battalova A., Bulk L., Nimmon L. (2020). I can understand where they’re coming from: how clinicians’ disability experiences shape their interaction with clients. *Qualitative Health Research*.

[26] Antonelli J., Jones S. J., Burridge A. B., Hawkins J. (2020). Understanding the self-regulated learning characteristics of first-generation college students. *Journal of College Student Development*.

[27] Morris T. H. (2020). Experiential learning – a systematic review and revision of Kolb’s model. *Interactive Learning Environments*.

[28] Damianakis T., Barrett B., Archer-Kuhn B., Samson P. L., Matin S., Ahern C. (2020). Transformative learning in graduate education: masters of social work students’ experiences of personal and professional learning. *Studies in Higher Education*.

